The article "Construction and evolutionary factors of spatial correlation network of China's provincial tourism resource conversion efficiency" was retracted in 2025. Reasons: unreliable results or conclusions; concerns about the citations.

# Construction and evolutionary factors of spatial correlation network of China's provincial tourism resource conversion efficiency

**DOI:** 10.1016/j.heliyon.2024.e28740

**Published:** 2024-03-31

**Authors:** Zhenjie Liao, Shan Liang

**Affiliations:** a School of Management, Guangzhou Huashang College, Guangzhou, 511300, China; b School of Economics, Guangzhou City University of Technology, Guangzhou 510800, China

**Keywords:** Tourism resource conversion efficiency, Network structure, Social network analysis, Block model analysis, China

## Abstract

**Research objective:**

To explore the spatial correlation network characteristics and formation mechanisms of tourism resource conversion efficiency, and provide reference for the collaborative improvement of tourism resource conversion efficiency at the provincial level in China.

**Research methods:**

Non parametric SBM efficiency measurement method and social network analysis method. Research hypothesis: The spatial network correlation characteristics of tourism resource conversion efficiency are obvious, and regional connections are close.

**Research findings:**

(i) during the research period, the spatial connection strength of China's tourism resource conversion efficiency continued to increase and the spatial network structure of tourism resource conversion efficiency tended to become more complex and significantly more stable. (ii) A spatially linked network with a stable tourism resource conversion efficiency structure formed in China. The number of network relations and density of the network fluctuated and increased, while the network efficiency continued to decrease; however, a strong small-world nature was observed. (iii) The economic development level difference matrix, tourism industry agglomeration difference matrix, human capital difference matrix, and marketization degree difference matrix significantly and positively affected spatial association relationship establishment, while the provincial adjacency matrix significantly and negatively affected such relationships.

## 1 Introduction

The extensive growth characteristics of China's tourism industry have been obvious for a number of years; however, the quality and quantity of the development trends are inconsistent. The allocation of tourism resources lacks rationality, which has caused serious resource waste [1]. Therefore, improving tourism efficiency and pursuing sustainable development have become foci of attention in the academic community in recent years. As the status of the tourism industry has improved, the quality of tourism economic growth has also received attention from all sectors of society [2]. However, the relationship between the quality of economic growth is multifaceted, and methods of objectively and correctly measuring the quality of tourism economic growth must be identified. Scholars have attempted to construct a comprehensive evaluation system for economic quality in different dimensions [3]. Although the evaluations focus on different topics, economic efficiency is considered one of the important indicators [4]. Some scholars have adopted a narrow perspective and believe that the quality of economic growth can be measured by economic efficiency [5,6]. Early research on the efficiency of the tourism industry evaluated the operational efficiency of tourism-related enterprises, such as hotels, travel agencies, tourism transportation companies, and museums, from the perspectives of management efficiency and operational efficiency [[7], [8], [9]]. Subsequently, the research content continued to enrich, including the ecological efficiency, resource efficiency, water use efficiency, poverty alleviation efficiency, supply chain efficiency, etc. of tourism [[10], [11], [12]].

The tourism industry plays an important role in promoting stable economic development; therefore, it has received increasing attention. Moreover, research on tourism efficiency is also becoming increasingly popular. Research on the efficiency of the tourism industry has been performed from various perspectives, such as the factors that influence tourism efficiency and the methods of evaluating tourism efficiency [13]. First, in terms of research content, the main focus is on the study of spatial characteristics [14], regional differences [15], evolution processes [16], influencing factors [17], and other issues. The research scale mainly focuses on countries, provinces, urban agglomerations, and cities [[18], [19], [20], [21]]. Among them, research on tourism efficiency in provinces is the most typical. In terms of the factors that affect tourism efficiency, scholars have focused on technological innovations, government regulations, institutional changes [22,23], modern service industry agglomeration, economic development level, tourism industry structure, degree of openness to the outside world, and transportation convenience [24,25]. Finally, mainstream comprehensive evaluation methods for tourism efficiency include the DEA, Malmquist index, and stochastic frontier analysis methods [26]. The efficiency of tourism resource conversion affects the comprehensive income of the tourism industry and also reflects the technological connotation of tourism industry development. Improving the efficiency of tourism resource conversion is a prerequisite for high-quality development of the tourism economy. However, a clear definition of the efficiency of tourism resource conversion has not been postulated. Therefore, this article defines the efficiency of tourism resource conversion as the comprehensive income obtained based on units of tourism resource supply at a certain technological level. At present, research on the efficiency of the tourism industry mostly focuses on the comprehensive efficiency of tourism industry development, while research on the conversion efficiency of tourism resources as an input factor is lacking. As a result, the conversion efficiency and mechanism of tourism resources remain a black box.

Based on the existing literature, it can be concluded that the analysis of the spatial correlation network and its formation mechanism of tourism resource transformation from a networked perspective is still relatively weak. Although some literature has verified the spatial spillover effect of tourism resource conversion efficiency based on geographical proximity relationships [27], it is mainly limited by the spatial quantification of attribute data, making it difficult to accurately characterize the spatial correlation network structure and evolution characteristics of tourism resource conversion efficiency [28]; At the same time, with the promotion of regional coordinated development strategy and marketization, the spatial correlation between regions is increasingly presenting a complex network structure, which provides a practical basis for analyzing the evolution characteristics and impact mechanisms of the spatial correlation network structure of tourism resource conversion efficiency from the perspective of complex networks and based on “relationship data” [[29], [30], [31], [32]]. Social Network Analysis (SNA), as an interdisciplinary analysis method, can use “relational data” to comprehensively analyze the spatial correlation network and its structure of a system, effectively overcoming the shortcomings of “attribute data” [33,34]. In recent years, it has been widely applied in the study of complex regional correlation networks, but few scholars have applied it to the theme of tourism resource conversion efficiency research.

In view of this, the study builds upon previous research results [35], analyzes the evolution characteristics and influencing factors underlying the spatial correlation network structure of China's tourism resource conversion efficiency from the perspective of complex networks, thereby providing insights for the study of green development in the tourism industry from a geographic perspective. Compared to existing research, the possible marginal contributions in the article include the 1) research perspective, in which “relational data” based on a relational perspective are used to explore the spatial correlation relationship of China's tourism resource conversion efficiency, accurately identifying the roles and positions of each region in the spatial correlation network; 2) research methods, in which the SBM-DEA model is used to effectively eliminate the influence of environmental factors and random disturbances and accurately measure the efficiency of tourism resource conversion and the QAP method is used to accurately identify the driving factors of the spatial correlation network of China's tourism resource conversion efficiency; and 3) research contents, in which the spatial correlation network structure characteristics and driving factors of tourism resource conversion efficiency are explored with a focus on China's provinces.

## 2 Study design

### 2.1 Measurement of tourism resource conversion efficiency based on modified DEA model

In 2001, Tone first proposed the SBM model based on unexpected outputs [36], and this method is widely used to measure the economic efficiency of multiple inputs and outputs in evaluation units. This model can comprehensively evaluate regional economic efficiency from both expected and unexpected perspectives, thereby effectively solving the problem of congestion or relaxation in various input-output units caused by radial and angular factors in traditional DEA models. However, the SBM model has a common problem with traditional DEA models, which is that it cannot effectively distinguish results with an efficiency of 1 for all evaluation units. Therefore, further analyzing the differences in efficiency values among each evaluation unit is difficult. In this context, Tone proposed the super efficiency SBM model, which combines the advantages of the super efficiency DEA model and SBM model and can effectively distinguish the evaluation units located at the forefront (efficiency value greater than 1) [37]. Therefore, this article adopts an output oriented super efficiency SBM model to measure the efficiency of tourism resource conversion in 31 provinces of China. The specific calculation formula is as follows [38]:

(1) $$\left\{ \begin{array}{c} \min_{p}=\frac{1+\frac{1}{m}\sum_{i=1}^{m}\frac{s_{i}^{-}}{x_{ik}}}{1-\frac{1}{q}\sum_{r=1}^{q}\frac{s_{r}^{+}}{y_{rk}}}\\ s.t.\sum_{j=1,j\neq k}^{n}x_{ij}\lambda_{j}-s_{i}^{-}\leq x_{ik}\\ \sum_{j=1,j\neq k}^{n}y_{rj}\lambda_{j}+s_{r}^{+}\geq y_{rk};\lambda_{j},s^{-},s^{+}\geq 0 \end{array}\right.$$

where *i* is the input index, with a range of [1, *m*]; *r* is the output indicator, with a value range of [1, *q*]; *ρ* represents the efficiency value of the evaluated DMU. *s*^−^ and *s*^+^ represent input and output relaxation variables, respectively; *λ* representing economies of scale; *k* refers to the evaluation DMU that has been removed from the *j*th index.

### 2.2 Feature characterization method for spatial correlation network structure of tourism resource conversion efficiency

Based on social network analysis, the overall characteristics, individual characteristics, and block models of the spatial correlation network of China's tourism resource transformation efficiency were studied [39]. This method is an interdisciplinary analysis method that uses mathematical methods and graph theory tools to explore the impact of relationship structures on structural components or the whole from the perspective of “relationships” [40]. It is currently widely used in network structure analysis in different fields. This article mainly uses four indicators to characterize the overall network characteristics of the spatial correlation of China's tourism resource conversion efficiency: network density, number of network relationships, network hierarchy, and network efficiency [41]. In addition, the following three centrality indicators are used to measure the position and function of each province in the development process of tourism resource conversion efficiency in the spatial network: point centrality, proximity centrality, and intermediary centrality [42]. This article takes the spatial connectivity mode of tourism resource conversion efficiency as the main thread. Based on grasping the overall characteristics of the spatial correlation network of tourism resource conversion efficiency, block models and model structure analysis methods are used to examine the spatial connectivity mode and its changes of tourism resource conversion efficiency from both macro and micro perspectives, and to identify the roles played by each region in the network. Through the analysis process from overall to partial and then to individual dimensions, this article attempts to systematically depict the spatial correlation characteristics of China's tourism resource conversion efficiency layer by layer. Table 1 presents the main indicators and their meanings used in this article to characterize the spatial correlation network characteristics of tourism resource conversion efficiency, which will be explained in detail below.

**Table 1:** Characteristic indicators of spatial correlation network structure for tourism resource conversion efficiency.

Indicator categories and names		Meaning of indicators
Overall characteristics	Average node degree	The average number of inter regional correlation relationships in the spatial correlation network of tourism resource conversion efficiency indicates the overall correlation strength of tourism resource conversion efficiency in the network.
	QAP correlation analysis	Identify the temporal evolution characteristics of the spatial correlation network of China's tourism resource conversion efficiency between different years.
Macro connectivity mode Micro connectivity mode	Block model Model structure	
		The same type of sector reflects the roles and patterns of each sector in the spatial correlation network of tourism resource conversion efficiency Identify the spatial correlation patterns of regional preferences in the spatial correlation network of tourism resource conversion efficiency through simulation

The block model is mainly used to identify the position and role of each node in the network through spatial clustering analysis. However, due to the different roles played by different plates composed of different regions in the network, we can determine the transmission mode of carbon emissions in the spatial correlation network by the correlation direction between plates According to the principle of block model, the roles played by each region in the network can be divided into the following four categories: 1) Bidirectional overflow plate, which has outgoing relationships with members within the plate and other plates, but less receiving relationships with other plates; 2) The main beneficiary sector has a higher degree of correlation among its internal members, but less external relationships, and receives relationships from other sectors, mainly characterized by “benefits”; When the number of receiving relationships from other sectors is much greater than the number of external sending relationships of the sector, or even when there are only receiving relationships but no external sending relationships, it can be called a net beneficiary sector; 3) The net overflow sector has a relatively small number of outgoing relationships with members within the sector, and also receives very few outgoing relationships from other sectors, mainly manifested as outgoing relationships with other sectors; 4) The brokerage sector has frequent receiving and sending relationships with other sectors, but there are fewer connections among members within the sector, playing a mediating role in promoting connections between different sectors This article will describe the different roles of the four types of plates mentioned above in the network through a string diagram.

### 2.3 Identification method of spatial correlation network formation mechanism for tourism resource conversion efficiency: QAP regression analysis

QAP is a non parametric testing method used to study the factors that influence relational networks [43]. QAP compares the values of each unit in the network matrix based on data permutation, obtains the correlation and regression coefficients between matrices, and conducts non parametric tests on the coefficients to avoid the “collinearity” problem caused by relational data regression [44]. Therefore, this article adopts the QAP regression analysis method to study the factors that affect the efficiency of the spatial correlation network transformation of tourism resources, in order to further reveal the formation mechanism of inter provincial correlations.

### 2.4 Indicator selection

#### 2.4.1 Setting of input-output factors for tourism resource conversion efficiency

Considering the rationality and consistency of the data, the number of travel agencies, hotels, tourism practitioners, tourism resources, and fixed asset investment are selected as input variables for the tourism industry. Among them, the number of travel agencies represents the service capacity of the tourism industry; the number of hotels represents the reception capacity of the tourism industry; the number of tourism practitioners represents the scale of tourism industry services; and fixed asset investment represents the scale of investment in the tourism industry. The number of tourists received and tourism income are used as output indicators, and they represent the tourism scale output and tourism economic output, respectively (see Table 2).

**Table 2:** Evaluation indicator system of tourism resource conversion efficiency.

Type	Indicator name	Indicator description
Input variables	Number of travel agencies	Tourism industry service capacity
	Number of hotels Number of tourism practitioners Fixed asset investment	Tourism industry reception capacity Scale of tourism industry services Investment scale of tourism industry
Output variables	Number of tourist receptions	Tourism scale output
	Tourism revenue	Tourism economic output

Using the year 2000 as the base period, the annual CPI index is used to deflate tourism income to eliminate inflation effects. By referencing the “Classification, Investigation and Evaluation of Tourism Resources” (GB/T18972-2017) and performing a literature review and field research, the entropy weight method was used to construct a tourism resource evaluation index system with three dimensions and 13 indicators, including comprehensive tourism resources, humanistic tourism resources, and natural tourism resources (see Table 3). The expert consultation method was used to screen and adjust the initially selected indicators and determine the weights of each indicator based on previous research findings [45]. If a resource is of multiple types, then the resource is only calculated based on the type with the highest weight value to avoid duplicate calculations.

**Table 3:** Tourism resource evaluation index system.

Target layer	Criterion layer	Indicator layer	Average weight
Tourist resources	Comprehensive tourism resources (0.4)	World Heritage (Double Heritage)	0.40
		5A level tourist attractions	0.35
		4A level tourist attractions	0.20
		3A level and below tourist attractions	0.05
	Humanistic tourism resources (0.3)	World Heritage (Cultural Category)	0.34
		National Intangible cultural heritage	0.16
		National Key Cultural Relics Protection Units	0.22
		National Historical and Cultural City	0.28
	Natural tourism resources (0.3)	World Heritage (Natural Category)	0.28
		National Nature Reserve	0.24
		National Forest Park	0.16
		National Urban Wetland Park	0.18
		National Geopark	0.14

#### 2.4.2 Factors affecting the efficiency of tourism resource conversion

Considering that the efficiency of tourism resource conversion is influenced by various factors such as macro and micro, and referring to existing literature [45], the following six factors are comprehensively selected. ① Economic development level (E). The level of economic development is the original driving force for improving the efficiency of tourism development. Improving infrastructure, introducing advanced technology, and innovating tourism products all require a certain amount of capital investment and are represented by the per capita GDP of each province. ② Traffic conditions (TA). Such conditions are an important factor affecting the development of the tourism industry because the spatial distribution of tourism resources in China is uneven. The ratio of highway mileage (km), railway mileage (km), and inland waterway mileage (km) to the area of each province (km^2^) and the ratio of takeoff and landing flights to the population of each province represent the development level of the four transportation modes, with the entropy weight method used for weighted summation. ③ Tourism industry cluster (CL). The spatial agglomeration and water balance of tourism industry elements are represented by the development scale of tourism industry in each region, and the tourism specialization of each province and city is used to determine the innovation capability (TP). It is generally believed that innovation capability has a positive promoting effect on the efficiency of the tourism industry. The entropy weight method is used to calculate the comprehensive scores for the total authorization of three types of patents, RD funding investments, and local financial science and technology funding in each province. ⑤ Human capital (HR). New growth theory postulates that knowledge and human capital are the “source” of innovation. Labor factor input is an important factor for promoting the development of the tourism industry, which is expressed by multiplying the number of people in various schools by the total number of years in various Educational stage. ⑥ Degree of marketization (MI). Usually, higher marketization can effectively allocate resources and improve resource conversion efficiency through competition mechanisms, pricing mechanisms, and supply and demand mechanisms.

### 2.5 Data sources

The data used in this study were sourced from the “China Tourism Statistical Yearbook” (2001–2021), “China Statistical Yearbook” (2001–2021), statistical yearbooks of various provinces, districts, and cities (http://www.stats.gov.cn), National Park Network (http://www.gjgy.com), China Cultural Heritage Bureau website (http://www.ncha.gov.cn), China intangible cultural heritage website (http://www.Nmchzg.com), and domestic airport production statistics bulletins (2001–2021). Due to data limitations, this study does not include the Hong Kong, Macao, and Taiwan regions.

## 3 Efficiency analysis

This article is based on DEASOLVER Pro 5.0 software and uses non radial (non directional) and variable return on scale (VRS) super efficient SBM models to calculate the tourism resource conversion efficiency of 31 provinces and cities in China from 2000 to 2020. The annual average value is estimated, and the usual 11:8:12 east-west regional division method is used. A comparative analysis was conducted on the conversion efficiency of tourism resources in different regions (Fig. 1).

**Fig. 1:** The evolutionary trend of tourism resource conversion efficiency in China from 2000 to 2020.

Using the non-parametric kernel density function of normal Gaussian distribution, we continue to explore the clustering difference of tourism resource conversion efficiency over time among provinces and cities. Taking the years 2000, 2005, 2010, 2015 and 2020 as observation time points for the estimation of nuclear density, the distribution of nuclear density at different time points was obtained (Fig. 2).

**Fig. 2:** Spatial correlation network of China's tourism resource conversion efficiency.

## 4 Network structure characteristics analysis

### 4.1 Overall characterization

A spatial correlation network was constructed based on the spatial correlation matrix of China's tourism resource transformation efficiency from 2000 to 2002. Due to space limitations, this article selected five cross-sections from 2000, 2005, 2010, 2015, and 2020, and visualized them using ArcGIS software, as shown in Fig. 2. The figure shows that the number of affiliations varies significantly among provinces. Shanghai, Beijing, Tianjin, and Zhejiang have established more affiliations with other provinces, with Shanghai firmly occupying the top position by establishing affiliations with 29 provinces in 2000, 2005, 2010, 2015, and 2020 and Hebei, Inner Mongolia, and Shanxi establishing fewer affiliations with other provinces. At the same time, the number of associated relationships in the eastern region is generally greater than that of the central, western, and northeastern regions. The number of relationships in the eastern region in 2020 accounted for 50.368% of the overall relationships, which was related to the developed tourism economy and better ecological environment in this region.

In order to further characterize the overall structural characteristics of the annual spatial correlation network, this paper used Ucinet software to measure the structural characteristics of the annual relationship number, network density, network correlation, network efficiency, and network hierarchy, as shown in Fig. 3, Fig. 4.

**Fig. 3:** Spatial correlation network density and network relationship.

**Fig. 4:** Spatial correlation network efficiency and network hierarchy.

In this paper, we build a stochastic network of the same size and density as the real correlation network each year, and use CCA, APLActal, CC random, and APL stochastic to represent the agglomeration coefficient and average path length of the real correlation network and the stochastic network, as shown in Fig. 5. The overall aggregation coefficient of the network is relatively stable, and the average path length fluctuates greatly. For example, CCratio/APLratio fluctuates between 1.097 and 3.108 per year, and in recent years, the average path length has increased due to the increase in network relationships, and the value of 1.097–3.108 has shown a downward trend. However, these values are all greater than 1, suggesting that the annual spatial connectivity network has a strong small-world feature [46,47]. In addition, the network connectivity is good, and the regions can also use the existing network structure to realize the rapid flow of resources and improve the efficiency of the transformation of tourism resources. However, with the gradual improvement of the tourism network, all provinces should find redundant channels to continuously improve the efficiency of tourism resource transformation.

**Fig. 5:** Evolution of small world characteristics of spatial correlation network.

### 4.2 Analysis of individual characteristics

The Ucinet software has been used to measure the degree centrality, intermediate centrality, and proximity centrality of spatial association networks in 2020, as shown in Table 4.

**Table 4:** Individual characteristics of spatial correlation network of China's tourism resource conversion efficiency in 2020.

Order	Province	Degree Centrality			Betweenness	Proximity to the center	
		In-Degree	Out-degree	Degree Centrality		In-Closeness	Out-Closeness
1	Beijing	28	5	93.333	25.087	33.333	93.75
2	Tianjin	26	4	86.667	62.393	37.975	73.171
3	Hebei	12	2	40	1.232	34.091	41.667
4	Shanxi	16	2	53.333	3.543	34.884	56.604
5	Inner Mongolia	11	2	36.667	0.148	34.884	36.585
6	Liaoning	13	2	43.333	0.725	34.884	40
7	Jilin	20	3	66.667	0.148	41.667	36.585
8	Heilongjiang	11	2	36.667	0.583	34.091	40
9	Shanghai	28	5	93.333	119.179	37.975	93.75
10	Jiangsu	27	4	90	224.007	41.096	90.909
11	Zhejiang	24	4	80	6.775	33.708	73.171
12	Anhui	12	2	40	0.805	34.091	54.545
13	Fujian	22	4	73.333	0.148	31.579	75
14	Jiangxi	11	2	36.667	1.268	33.708	54.545
15	Shandong	28	5	93.333	108.657	48.387	54.545
16	Henan	14	2	46.667	21.446	36.585	57.692
17	Hubei	26	4	86.667	9.991	46.875	38.961
18	Hunan	17	3	56.667	5.627	35.294	60
19	Guangdong	23	4	76.667	8.944	33.708	71.429
20	Guangxi	20	3	66.667	13.419	36.145	62.5
21	Hainan	16	2	53.333	6.41	34.884	58.824
22	Chongqing	19	3	63.333	25.034	37.5	57.692
23	Sichuan	14	2	46.667	13.002	34.483	58.824
24	Guizhou	11	2	36.667	5.539	37.037	56.604
25	Yunnan	23	4	76.667	63.939	42.857	56.604
26	Tibet	7	1	23.333	0.148	29.412	40.541
27	Shaanxi	13	2	43.333	0.771	32.967	57.692
28	Gansu	11	2	36.667	0.503	32.258	57.692
29	Qinghai	10	1	33.333	0.764	32.258	58.824
30	Ningxia	11	2	36.667	0.764	32.258	60
31	Xinjiang	28	5	93.333	0	93.75	3.226

Intermediate centrality can be used to measure the degree of intermediary role of each province in the network, thus reflecting the ability to control resources. The differences in intermediate centrality were obvious, with the maximum difference reaching 22.673. Shanghai and Jiangxi were in the top two and had much larger values than the other provinces. This finding indicates that the above-mentioned areas are mostly in the middle of the exchange between nodes, play an important “bridge” role, and show a stronger control over resources. Beijing, which ranked second in terms of degree centrality, was in the sixth place in terms of intermediate centrality. This shows that although Beijing is associated with more provinces, its intermediary role is relatively small and it has more of a beneficiary effect in the network. It is worth noting that Xinjiang, Ningxia, Inner Mongolia, and other regions are located in remote areas, the intermediate centrality of these areas is 0, and they do not play a mediating role in the network. Inner proximity centrality refers to the ability of a node to influence other nodes, Shanghai, Beijing, and Zhejiang were in the top three and had the greatest influence on the efficiency of the tourism resource conversion in other provinces, which is mainly due to their superior location conditions. Corresponding to the internal proximity to the center degree, the external proximity to the center degree refers to the degree of influence of a node refers to other nodes, Liaoning, Xinjiang, and Ningxia ranked at the top, indicating that the tourism resource conversion efficiency of the above regions are influenced by neighboring or non-neighboring provinces to a greater extent. This finding reflects the remote location of the region, which led to fewer affiliations and relatively singular sources of resources. Thus, tourism resource conversion efficiency is highly susceptible to the influence of associated provinces.

### 4.3 Block mold analysis

The above analysis clearly shows that each province's position and role in the network is different, showing significant regional differences. In order to further reveal the role of each region in the network and describe the interaction between regions, based on the spatial correlation network of tourism resource conversion efficiency in 2020, China is divided into four regions by using the CONCOR algorithm of Ucinet software. The results are shown in Table 5.

**Table 5:** Division of spatial correlation network of China's tourism resource conversion efficiency.

Section	Section matrix				Relation-ships	Acceptance	Expectation （%）	Actual （%）	Characte-ristics
	1	2	3	4					
1	15	16	44	8	15	26	57.69	42.30	Main overflow
2	20	28	19	9	28	10	35.71	34.28	Main overflow
3	36	12	5	2	5	57	8.77	27.41	Main overflow
4	8	10	24	7	7	31	22.58	1.29	Brokers

There are 15 internal relations and 26 external acceptance relations in plate I, and the proportions of expected and actual internal relations are 57.69% and 42.30%, respectively, this indicates that the plate has more external spillovers and less internal spillovers and can be classified as a major spillover plate [48]. The internal coefficient of plate II is 28, and the external acceptance coefficient is 10. The proportion of expected and actual internal relations were 35.71% and 34.28% respectively. Therefore, this plate has more external spillover relationships, which can also be classified as a major spillover plate. Most of the provinces in plate I and II are located in the Midwestern Sectional Figure Skating Championships, with relatively backward economy and poor ecological environment, but rich in tourism resources. However, under the influence of external spillover, “Siphon effect” appears in the eastern developed areas. The internal coefficient of plate III is 5 and the external acceptance coefficient is 57. The proportion of expected and actual internal relations are 8.77% and 27.41% respectively, and the inter-plate relations are much larger than the spillover relations; therefore, they can be divided into the main beneficial sectors. The internal coefficient of the fourth plate is 7 and the external acceptance coefficient is 31. The proportion of expected and actual internal relations were 22.58% and 1.29% respectively. In addition, fewer connections are observed outside the plate, and more acceptance and spillover relationships are observed. As a result, these relationships are more balanced and assume a greater“Bridge” role. Therefore, this sector can be classified as the brokerage sector. In the future, the fourth plate should strengthen internal links. In order to show the spillover relationship between plates, the density matrix within and between plates in 2020 is measured, the class matrices within and between plates are measured based on the overall density of the correlation network (0.194) (Table 6).

**Table 6:** Efficiency density matrix and image matrix of China's tourism resource conversion efficiency.

Section	Density matrix				Image matrix			
	Section 1	Section 2	Section 3	Section 4	Section 1	Section 2	Section 3	Section 4
Section 1	0.75	0.938	0.944	0.6	1	0	0	0
Section 2	0.25	0.667	0.625	0.65	0	0	1	0
Section 3	0.417	0.028	0.059	0.9	0	1	0	1
Section 4	0.2	0.05	0.022	0.55	1	0	1	0

Overall, the spatial relationship of China's tourism resource transformation efficiency mostly occurs between sectors, with relatively loose intra sector relationships and relatively strong inter sector relationships. It is necessary to strengthen the connections between provinces in the sector. In addition, the roles of each sector in the network are also heterogeneous. Plate 1 and plate 2 are the main spillover sectors with more spillover relationships, plate 3 is the main beneficiary sector, and plate 4 is the intermediary sector, playing an important intermediary role.

## 5 QAP regression analysis

### 5.1 Selection of indicators

This paper selects the geographical distance between provincial capitals, and considers whether the provincial capitals are adjacent as one of the factors affecting the spatial correlation network. The analysis of block model shows that the interaction between plates is related to the level of economic development, and more plates show more developed economic and spillover relationships. In addition, social and economic factors such as traffic conditions, tourism industry agglomeration, innovation ability, human capital and marketization degree will also have an impact on the network structure of tourism resource conversion efficiency [49]. Therefore, this paper takes the above indicators as influencing factors. And the following model is constructed:

*N*_*i*_ = *f* (*D, W, E, TA, CL,TP, HR, MI*)

In the formula, *Ni* represents the spatial correlation network for the *i*th year; *D* represents the geographic distance matrix between capital cities; *W* represents the provincial adjacency matrix, where the adjacency matrix is 1 and the non adjacency matrix is 0; *E* is the matrix of economic development level differences, measured by provincial GDP; *TA* represents the matrix of differences in transportation conditions, and it is measured by the level of development of the four modes of transportation in each province; *CL* represents the differentiation matrix of tourism industry agglomeration, and it is measured by the level of tourism specialization in each province; *TP* represents the innovation capability difference matrix, and it is measured by the comprehensive scores of the total number of three types of patent authorizations, RD funding investment, and local financial science and technology grants in each province; *HR* represents human capital, and it is measured by the number of college students in each province; and *MI* represents the difference matrix of marketization degree, and it is measured by the marketization index of each province. Select 5000 randomly arranged tourism resources using Ucinet software to obtain the spatial correlation matrix of tourism resource conversion efficiency. The correlation coefficients of various influencing factors in 2000, 2005, 2010, 2015, and 2020 are shown in Table 7.

**Table 7:** Correlation analysis.

Variable	2000	Significance	2005	Significance	2010	Significance	2015	Significance	2020	Significance
*E*	0.852**	0.012	0.552*	0.022	0.152*	0.042	0.764**	0.013	0.214*	0.022
*TA*	0.474**	0.024	0.133*	0.042	0.723	0.013	0.334	0.034	0.262	0.014
*CL*	0.172	0.045	0.721	0.011	0.314	0.034	0.893**	0.012	−0.173*	0.033
*TP*	0.776	0.013	0.264	0.033	0.865***	0.013	0.542	0.023	0.024	0.094
*HR*	0.348**	0.034	0.833**	0.015	0.466	0.024	0.433*	0.124	0.115*	0.054
*MI*	0.883	0.012	0.392	0.024	0.187*	0.053	0.531	0.525	−0.113*	0.052
*D*	0.271*	0.187	0.312	0.143	−0.063	0.498	−0.102*	0.378	0.173	0.252
*W*	−0.512	0.042	−0.561**	0.03	0.421*	0.079	0.459*	0.061	−0.612**	0.022

Note: * indicates p < 0.1, * * indicates p < 0.05, and * * * indicates p < 0.01. The same below.

### 5.2 Regression analysis

Based on the model, the spatial correlation matrix of China's tourism resources transition efficiency and its influencing factors in 2000, 2010 and 2020 were analyzed by using Ucinet software. We selected 5000 random permutations, and the regression results are shown in Table 8. The adjusted *R*^2^ values were 0.441, 0.531, 0.631 respectively, which passed the 1% significance test. This finding suggests that changes in these factors may better explain changes in spatial correlation. The regression coefficients of the geographical distance matrix in 2000, 2010 and 2020 were 0.635, −0.271, −0.382 respectively, indicating that the smaller the geographical distance between provinces, the more favorable it is to establish spatial correlation. The regression coefficients of the difference matrix of economic development level in 2000, 2010 and 2020 are 0.323, 0.583 and 0.734 respectively, passing the significance test at the levels of 10%, 1% and 5% respectively, and the coefficients are positive, reflecting the widening gap of economic development level among regions, which is conducive to the establishment of spatial correlation between regions. The regression coefficients of the tourism industry agglomeration difference matrix in 2000 and 2020 are 0.388 and 0.721 respectively, passing the significance test at the level of 5% and 10% respectively, and the coefficients are positive, reflecting the increasing level gap of industrial agglomeration difference between regions, which is conducive to the establishment of spatial correlation between regions. The regression coefficients of human capital difference matrix in 2010 and 2020 are 0.741 and 0.649 respectively, passing the significance test at the level of 10% and 5% respectively, and the coefficients are positive, indicating that the greater the human capital difference, the more conducive to the establishment of correlation relationship. The regression coefficients of the marketization degree difference matrix in 2000 and 2010 are 0.043 and 0.543 respectively, passing the significance test at the level of 10% and 5% respectively, and the coefficient is positive, indicating that the greater the difference in marketization degree, the more conducive to the establishment of spatial relations. Provinces with higher marketization degree have more frequent interactions with foreign enterprises, universities and scientific research institutions. It can receive a large number of foreign innovation resources, which is more attractive to domestic neighboring provinces with a low degree of openness, and is conducive to the establishment of interactive relations.

**Table 8:** QAP regression analysis.

Variable	2000			2010			2020		
	Coefficient	Probability1	Probability2	Coefficient	Probability1	Probability2	Coefficient	Probability1	Probability2
*E*	0.323*	−0.072	0.115	0.583***	0.433	0.012	0.734**	0.324	0.032
*TA*	0.032	0.023	0.016	0.875	0.655	0.024	0.604	0.874	0.016
*CL*	0.388**	−0.054	0.092	0.687	0.215	0.045	0.721*	0.454	0.022
*TP*	0.043	0.008	0.013	0.522	0.783	0.018	0.674	0.188	0.042
*HR*	0.424	−0.033	0.094	0.741*	0.355	0.037	0.649**	0.786	0.018
*MI*	0.043*	0.013	0.014	0.543**	0.921	0.014	0.601	0.355	0.032
*D*	0.635	0.831	0.376	−0.271	0.579	0.759	−0.382*	0.872	0.482
*W*	−0.378	0.921	0.482	0.789	0.374	0.671	−0.483	0.657	0.723
*Adj R*^2^	0.441	−0.057	0.126	0.531**	0.565	0.026	0.631	0.905	0.014
*Sample size*	482			482			482		

## 6 Conclusion and discussion

### 6.1 Conclusion

This article uses an efficient SBM model to calculate the efficiency of tourism resource transformation in 31 provinces of China from 2000 to 2020. Based on this, an improved gravity model is used to construct a spatial correlation network for the efficiency of tourism resource transformation in China, and the network structure is analyzed. Then, through QAP regression analysis, the factors affecting the spatial correlation network were studied, and the following conclusions were drawn.

Firstly, from the perspective of network structure characteristics, the overall feature analysis indicates that all provinces have established interactive relationships with neighboring or even non neighboring provinces, indicating that China has formed a relatively stable spatial correlation network for tourism resource conversion efficiency. The number of network relationships and density fluctuate, the hierarchy and efficiency of the network decrease, and the number of redundant channels connecting nodes increases. However, the network still has a strong small world nature, and regions should strengthen the identification of redundant channels to further improve the efficiency of resource dissemination.

Secondly, from the perspective of network centrality, through the analysis of individual characteristics, we have discovered a clear network core edge structure. Provinces and cities such as Shanghai, Beijing, Zhejiang, and Jiangsu are located at the center of the network and play important intermediary roles due to their significant geographical advantages and greater connections with other provinces. However, Tibet, Xinjiang, Ningxia, Inner Mongolia and other provinces are at the edge of the network due to their remote location and lack of contact with other provinces. It can be seen that the conversion efficiency of tourism resources is easily influenced by other provinces.

Thirdly, from the perspective of the composition and function of the location members of each regional plate, the block model analysis shows that the spatial correlation network of China's tourism resource transformation efficiency has formed four major plates, with sparse inter plate connections, close inter plate connections, and strong spillover effects. The role of each sector in the network is heterogeneous. The developed eastern region, as the main beneficiary sector, has a significant “siphon effect” and benefits significantly. The central and western regions, as the main spillover sectors, generally show a significant spillover effect, while the southeastern coastal regions, as intermediary sectors, show a significant spillover effect.

### 6.2 Discussion

The social network analysis indicated that there is a significant spatial correlation between the conversion efficiency of tourism resources in China, which is consistent with the research findings of Cheng [43]. However, the overall network feature analysis revealed that the spatial correlation of the network was relatively low. The formation of spatial correlation networks was conducive to improving the efficiency of tourism resource conversion and promoting green and coordinated development of regional tourism industry. Local governments should focus on ecological environment protection and high-quality development strategies for the tourism industry, strengthen the coordination of relevant policies, design reasonable policies to smooth the circulation channels of tourism production factors, and create more spillover paths. Based on the above findings, the following recommendations have been provided to promote the overall improvement in the efficiency of China's tourism resource conversion.

(1) The supply side structural reform of tourism resources should be continuously promoted. Each province should scientifically and reasonably plan the scale and structure of the tourism industry according to local conditions, the consumption needs of tourists, and its own tourism resource advantages; optimize the allocation of tourism resources; develop new tourism products with strong participation, significant uniqueness, and high profit added value; increase the technological content of tourism resources; and achieve maximum marginal benefits of tourism resources.
(2) The market allocation of tourism resources should be increased by adhering to market-oriented reform, improving the property rights system and market-oriented allocation of factors, optimizing the allocation of tourism resources, reducing the government's discourse power in resource allocation, preventing blind increases in the number of tourism resources, and improving the efficiency of tourism resource conversion scale. Moreover, an environment for technological progress and independent innovation in tourism enterprises should be creased to enhance their initiative in independent innovation.
(3) The concept of coordinated development of global tourism should be strengthened. Each province should strengthen regional tourism cooperation, integrate tourism resources, coordinate overall planning, gather new resources for the development of regional tourism, promote the circulation of various production factors in tourism, expand the “penetration” and “multiplier” effects of the tourism industry, enhance the diffusion effect of technology, enhance the digestion ability of technology, establish an internal driving mechanism for technological innovation diffusion, and alleviate the efficiency differences in regional tourism resource conversion.

It should be noted that the above research also has the following shortcomings. First, due to the lack of data, the efficiency of tourism resource conversion under environmental constraints has not been considered. Second, at the national spatial scale, the non-equilibrium of tourism resource conversion efficiency gradually decreases. Therefore, whether there is “club convergence” within the eastern, central, and western regions must be determined. Moreover, future studies should focus on changes in tourism resource conversion efficiency at the provincial scale. Finally, the factors and mechanisms that affect the efficiency of tourism resource conversion among different types of tourism resources will differ. Classifying and studying the efficiency of tourism resource conversion among different types of tourism resources represents an important future research direction.

## Ethical approval and consent to participate

The authors declared that they have no known competing financial interests or personal relationships, which seem to affect the work reported in this article. We declare that we have no human participants, human data, or human issues.

## Funding

This study received support from the following sources: a grant from the Guangzhou Huashang College (No. 2022HSKT02); a grant from the Guangzhou Huashang College (No. 2021HSXK10); the Philosophy and Social Sciences of Guangzhou in the 14th Five-year Period (2023GZGJ314); a grant from the Guangzhou Huashang College (No. 2022HSDS22).

## Consent for publication

We do not have any individual person's data in any form.

## Data availability

Data will be made available on request.

## CRediT authorship contribution statement

**Zhenjie Liao:** Writing – review & editing, Writing – original draft, Formal analysis, Conceptualization. **Shan Liang:** Writing – review & editing, Writing – original draft, Software, Data curation.

## Declaration of competing interest

The authors declare that they have no known competing financial interests or personal relationships that could have appeared to influence the work reported in this paper.
